The article "Platypnea–Orthodeoxia Syndrome: Multiple Pathophysiological Interpretations of a Clinical Picture Primarily Consisting of Orthostatic Dyspnea" was retracted in 2021. Reason: duplicate publication.

# Platypnea–Orthodeoxia Syndrome: Multiple Pathophysiological Interpretations of a Clinical Picture Primarily Consisting of Orthostatic Dyspnea

**DOI:** 10.3390/jcm5100085

**Published:** 2016-09-23

**Authors:** Renato De Vecchis, Cesare Baldi, Carmelina Ariano

**Affiliations:** 1 Cardiology Unit, Presidio Sanitario Intermedio “Elena d’Aosta”, ASL Napoli 1 Centro, 80137 Napoli, Italy; carmelariano@tiscali.it; 2 Heart Department, Interventional Cardiology, Azienda Ospedaliero-Universitaria “San Giovanni di Dio e Ruggi d’Aragona”, 84131 Salerno, Italy; giovenale80@gmail.com

**Keywords:** platypnea, intracardiac shunts, ventilation/perfusion mismatch, pulmonary arteriovenous shunts

## Abstract

Platypnea–orthodexia syndrome (POS) is often a challenging diagnostic problem. It is characterized by dyspnea that is accentuated by standing or sitting positions due to a marked fall in blood oxygen saturation, and instead is improved by assuming the lying position. In the present brief review, the authors address the pathophysiology of POS, and outline its clinical symptoms as well as the main modalities of diagnostic evaluation and possible therapeutic options. Moreover, some problems concerning much-debated issues and persistent uncertainties about the pathophysiology of POS are presented along with the description of the diagnostic and therapeutic resources currently available for this syndrome.

## 1. Definition

Platypnea–orthodeoxia syndrome (POS) is distinguished by breathlessness that is alleviated when lying down and is exacerbated when sitting or standing up. It is the opposite of orthopnea and is characterized by a decrease in blood oxygen saturation in the passage from supine position to orthostatism [1,2,3,4]. 

Possible causes of this syndrome are intracardiac shunt, pulmonary parenchymal ventilation/perfusion mismatch, and pulmonary arteriovenous shunts. In Table 1, the main conditions that favor or elicit POS are listed. 

## 2. Pathophysiological Issues 

### 2.1. Cardiac POS

In the majority of cases, the syndrome is caused by the coexistence of an anatomical heart defect, especially patent foramen ovale (PFO), but also atrial septal defect (ASD) or atrial septal aneurysm (ASA) with septal fenestration, combined with structural or functional abnormalities of other thoracic or abdominal organs. Such an association is recognized as a critical factor capable of generating orthostatic dyspnea coupled with a fall in oxygen saturation that disappears in the recumbent position, i.e., the pathognomonic picture of this syndrome. For an insightful discussion on POS, it would be useful to make some logical considerations regarding the still poorly clarified aspects of the syndrome.

First of all, one should question why the oxygen desaturation is related to the orthostatism, and also why the syndrome mostly occurs in middle-aged or old people, although in the majority of cases, it is linked to a congenital defect in heart development (especially PFO, but also ASD or ASA with septal fenestration) that really dates from birth. In other words, PFO is present in 25% of the general population, according to autopsy studies [5]; however, it has been implicated in cryptogenic stroke in only a small minority of patients with this structural defect [6,7], while the cases in which PFO is manifested as a crucial anatomical factor in the genesis of POS are even less frequent, about 2% according to some authors [8]. It could be said that PFO exerts a clinically evident harmful influence, so as to generate the POS, only in the presence of other pathological conditions, e.g., aortic aneurysm, aortic elongation, pericardial effusion, pneumonectomy, etc. (see Table 1). Of course, most people with PFO never develop symptoms of POS because the left atrial pressure is 5–8 mmHg higher than the right atrial pressure and the atrial septum is functionally closed. Thus, this pressure difference is regarded as able to prevent right-to-left shunting through a PFO or small ASD in the majority of cases. However, right-to-left shunt can occur because of a flow phenomenon (anatomical distortion) and/or a transient pressure elevation in the right atrium (hemodynamic causes) [9,10,11,12] (see Table 1).

The most studied form of POS is the one caused by right–left shunt at the level of the atrial septum, so-called cardiac POS.

Indeed, a deformation of the atrial septum is usually present, and it plays a critical role in determining a change in the direction of blood flow that comes from venous caval orifices.

In these cases, a displacement of interatrial septum has been frequently demonstrated [9]; it affects the shape and the compliance of the right atrium, so that the atrial defect undergoes a change in its original position that puts it directly in line with the blood flow from the inferior vena cava at its entrance into the right atrium. This displacement is much more marked in upright posture, so as to promote an orthostatic preferential flow of desaturated blood through the area of septal discontinuity. This change in the axis of the atrial septum may be secondary to dilatation of the proximal ascending aorta [9,11] distorting the interatrial septum, a phenomenon that is probably exacerbated with age or by the existence of an associated aortic aneurysm (Figure 1 and Figure 2). Similar tilting of the septal atrium favoring the right-to-left atrial shunt through a preexisting defect may be observed after pneumonectomy [3]. 

Various anatomical and functional acquired causes have been documented in case reports regarding POS: for example, aortic aneurysmal dilation, paralysis and displacement in the chest of the right hemidiaphragm, both obstructive and restrictive pulmonary diseases, and skeletal abnormalities of the spine such as kyphoscoliosis [1,9]. These and other predisposing or precipitating conditions are listed in Table 1.

### 2.2. Ventilation/Perfusion Mismatch as Primary Cause of POS in Parenchimal Pulmonary Diseases and Pulmonary Arteriovenous Shunts

Besides cardiac POS, i.e., the most well-known type, there are other clinical phenotypes that depend on lung diseases that entail a ventilation/perfusion mismatch. In particular, idiopathic pulmonary fibrosis has been shown to have potential for generating POS. There are several case reports illustrating the causal relationship between diseases of the pulmonary parenchyma able to induce ventilation/perfusion mismatch, and the development of the typical clinical picture of POS (orthostatic dyspnea and fall of oxygen blood saturation, which regress by assuming the lying position).

Among these case reports, the article by Takhar et al. [13] refers to a case of POS combined with interstitial lung disease (ILD), where the existence of regional differences in pulmonary alveolar perfusion when comparing apical and basal regions of the lungs is strongly suspected. These regional discrepancies of respiratory function would not be uncommon in the presence of certain types of lung disease (in particular, interstitial lung fibrosis and viral or fungal pneumonia [14,15,16]) and would become more evident if the patients are asked to assume the upright position. The case described by Takhar et al. [13] refers to a middle-aged man with ILD who slumped onto the floor and whose oxygen saturation was subsequently examined with a pulse oximeter that showed marked hypoxia, which gradually recovered while he was supine on the floor. The constant occurrence of marked desaturation of the blood during even short periods (a few minutes) of upright or sitting posture was put in relation to a condition of marked ventilation/perfusion mismatch caused by the so-called diffuse zone 1 phenomenon. In this patient, there was a predominant basilar fibrosis of the lungs with relatively preserved apical segments. In healthy individuals, in standing position, the apical portion of the lung, termed as zone 1, remains hypoperfused during most of the cardiac cycle, except for flushes of blood during the peak ejection phase of systole. The lying position places more of the lung in zone 3 and virtually eliminates zone 1. In our patient, the basal parts of both lungs were predominantly affected by the disease, i.e., the fibrosis showed severe involvement of only those segments that in normal individuals have better perfusion and ventilation compared with apical regions. As a consequence, it is possible that when the described patient was in supine position, all the underperfused upper part of the lung (zone 1) converted in zone 3 leading to equal ventilation and perfusion, and ultimately adequate oxygenation. By contrast, whenever the patient was in the standing position, increased perfusion of the poorly ventilated diseased lower zone presumably elicited a marked ventilation/ perfusion mismatch leading to platypnea–orthodeoxia. This kind of explanation has also been used by other authors for similar cases [14,15,16]. 

Another cause of POS can be a flow of desoxygenated blood through arteriovenous shunts mostly in the bases of the lungs. The increased blood flow through the basilar regions in standing position increases the shunts and generates symptoms. This phenomenon is mostly observed in patients with hepatopulmonary syndrome (HPS). 

The term HPS is used to define the association of liver disease (usually liver cirrhosis), intrapulmonary vasodilatation at the capillary and precapillary levels, and impaired arterial oxygenation [17]. Although found most commonly in the setting of cirrhosis, HPS may occur across the spectrum of etiologies of liver disease, regardless of the presence of porto-pulmonary hypertension [18]. In addition, advanced liver disease is not required for HPS to develop, and the disease may worsen irrespective of hepatic function. Increased endogenous nitric oxide (NO) production appears to be the key priming factor for the development of pulmonary vascular dilatation. Although NO levels in the exhaled air of patients with HPS are increased, consistent with pulmonary overproduction, normalization has been observed after liver transplantation [19]. Regardless of the precise pathogenetic mechanism, pulmonary vascular dilatation allows the rapid or direct passage of poorly oxygenated mixed venous blood into the pulmonary veins. Characteristic (but not pathognomonic) features include platypnea and orthodeoxia, resulting from a gravitational increase in blood flow through dilated vessels in the lung bases. POS occurs in this case because the amount of dilated vessels is larger in the basal segments of the lungs; thus, orthostatism re-directs a considerable part of blood flow toward the basal segments of the lungs, thereby increasing the hematic volume that escapes from the alveoli and is excluded by effective respiratory exchanges.

## 3. Epidemiology 

POS is a rare condition. Indeed, its true prevalence in the population is not known. In addition, for a number of patients with POS, varying between 13% and 47% depending on different authors, the etiology cannot be identified with certainty, i.e., orthodoexia occurs without identifiable lung or heart disease [4,20,21]. A review of studies published in 2012 found 105 articles with a total of 188 patients, each of whom had received the diagnosis of platypnea and orthodeoxia [4]. 

## 4. Clinical Picture

Patients with POS suffer from dyspnea and/ or hypoxemia that arises in the upright position and is also present in the sitting position. These symptoms are usually attenuated or disappear within a few minutes by assuming a lying position [1,2].

The patients do not respond to traditional therapies for chronic lung disease, coronary artery disease or left ventricular dysfunction. Reports in the literature show that patients with POS have different adjunctive symptoms: tachycardia, tachypnea, decrease in systolic blood pressure in the upright position [12], and non-response to oxygen supply in the upright position [10]. 

## 5. Diagnostic Assessment

The initial assessment should be the evaluation of a possible association between breathlessness and upright position (Table 2). For this purpose, measurement of oxygen saturation and blood gas analysis (pulse oximetry) should be performed both in supine and upright positions; the presence of orthostatic desaturation should primarily direct the diagnosis toward an atrial septum discontinuity [4].

In HPS, a decrease in the partial arterial pressure of oxygen in the upright position of about 5% or at least 4 mmHg was assumed as a typical, although not patognomonic, feature [21]. One author notes that intracardiac shunting is not presented with clear postural changes in blood oxygenation in all patients. Supplemental oxygen therapy may provide support for diagnosing POS because the right-to-left atrial shunt prevents systemic oxygen saturation from reaching 100% [9].

Doppler-echocardiography and contrast-enhanced echocardiography are paramount for making the diagnosis. Both examinations should ideally be executed with the patient in lying position and upright position. These investigations may allow one to identify and localize the shunt at the atrial level because of the passage of microbubbles to the left atrium in the first three beats after opacification of the right chambers. Notably, in a few cases, the shunt can be seen only during a Valsalva maneuver [20]. In a review of the literature, Rodrigues et al. [4] found evidence that transthoracic contrast-enhanced Doppler echocadiography is possibly just as effective as transesophageal echocardiography [22]. If an intracardiac shunt is not confirmed, an intrapulmonary shunt can exist. In this case, the suggested image techniques, judged suitable for detecting intrapulmonary vascular dilatations, are contrast-enhanced echocardiography, perfusion scan (scintigraphy) with macroaggregated albumin and pulmonary arteriography [21]. Contrast-enhanced echocardiography is the most sensitive diagnostic tool, and, moreover, is less invasive than pulmonary arteriography. As opposed to an intracardiac communication, in HPS, the passage of microbubbles during contrast-enhanced echocardiography through the dilated pulmonary vessels to the left atrium shows a delay of three to six heart beats [4,21]. 

## 6. Treatment

Treatment depends on the cause of POS. In cases of intracardiac communication without pulmonary hypertension, closure of the defect is a causative therapy with a quick relief of symptoms. Closure can be surgical or percutaneous [4,9,10,11]. Nowadays, the percutaneous approach with cardiac catheterization to close PFO is the preferred option. Coexisting anatomic defects such as aortic aneurysm, aortic elongation (Figure 1 and Figure 2), constrictive pericarditis, or myxoma, however, require surgical intervention [1,3,23]. Percutaneous closure of PFO or ASD can be performed with specific devices, such as the Amplatzer Septal Occluder or Amplatzer PFO Occluder. After closure, both the aortic and the peripheral oxygen blood saturations have to be monitored. Residual shunt can be identified by echocardiography. Anticoagulation with acetylsalicylic acid should last three months following implantation. Transcatheter closure results in immediately increased oxygen saturation in the upright position after the procedure. Platypnea completely regresses [9,10,11,22,23].

In pulmonary diseases (chronic obstructive pulmonary disease, idiopathic pulmonary fibrosis, etc.), underlying pulmonary disorders must be treated to improve ventilation–perfusion matching [13].

In patients with HPS, advanced liver disease is the cause of POS, and liver transplantation is the only causal therapy [24]. First-line management can be oxygen therapy, bed rest, salt restriction and diuretics. Transplantation improves blood oxygenation in 80% of patients, but severe hypoxemia is a leading cause of perioperative mortality [24].

## 7. Conclusions

POS is a rare syndrome, characterized by the emergence of a right-to-left shunt at the intracardiac or intrapulmonary level. The clinical picture is distinguished by shortness of breath that worsens on standing because of accentuation of oxygen desaturation, and instead improves, at least partly, with the lying position.

Shunting blood from the right to the left heart through an atrial septal defect (PFO, ASD or ASA with septal fenestration) is the most common cause of the disease. In these cases, percutaneous or surgical closure of the atrial septal communication is mandatory. In the majority of cases, additional anatomic changes are identifiable, which ultimately generate POS. These changes can follow lung surgery and malformations such as kyphoscoliosis, or are age-related. Sometimes, the triggering role of certain anatomical changes remains unclear. In recent years, increasing articles and case reports of POS have elicited the attention of physicians, who have acquired a greater awareness of POS and have become more accurate in diagnosing and treating patients with unexplained or paroxysmal dyspnea.

## Figures and Tables

**Figure 1:** (**A**) Chest roentgenogram in the posterior–anterior view reveals pronounced cardiomegaly with marked projection of the right mediastinal border (arrowheads). (**B**) Sagittal view of contrast-enhanced 64 slice computed tomography shows the enlarged aortic root (Ao), which is posteriorly expanded with compression of the atrial chambers and their septum. (**C**) In the intraoperative views obtained after sternotomy, the enlarged and elongated aortic root nearly reaches the diaphragm, and (**D**) manual lifting of the ascending aorta exposes the posteriorly compressed right atrium (RA). (LA = left atrium; PA = pulmonary artery.)

**Figure 2:** Transesophageal echocardiography with color Doppler at the level position showing a patent foramen ovale (PFO) behind the enlarged aortic root (Ao). (**A**) In the supine position, paradoxical right-to-left shunt through the PFO is transiently observed as only a stream. (**B**) In the sitting position, the shunt grows to a massive jet. (**C**) A continuous-wave Doppler recording shows that shunt flow is observed in the systolic phase, with a peak velocity of 0.86 m/s (asterisk) and a calculated pressure gradient of 2.9 mmHg. (LA = left atrium; RA = right atrium.)

**Table 1:** Possible causes of platypnea–orthodeoxia syndrome.

Underlying Anatomical or Functional Alteration	Pathophysiologic Mechanism	Accompanying Pathologic Condition
Intracardiac shunt PFO ASD ASA with fenestration	Transient right–left shunt without elevated right–left pressure gradient	Compression of RA by aortic dilatation, elongation or aneurysm Pericardial effusion or constrictive pericarditis Postpneumectomy ^1^ Eosinophilic endomyocardial disease Abnormally lying Eustachian valve or Chiari network RA myxoma RA lipomatosis hypertrophy Kyphosis
	Transient right–left shunt with elevated right–left pressure gradient	Pulmonary thromboembolism Idiopathic pulmonary hypertension Right hydrothorax Long duration lung disease causing pulmonary hypertension Postpneumectomy
Pulmonary diseases with ventilation/perfusion mismatch	High V/Q ratio	Emphysema COPD Interstitial lung disease
	Low V/Q ratio	Hepatopulmonary syndrome Pulmonary arteriovenous malformations or fistulae Rendu–Osler–Weber syndrome

PFO, patent foramen ovale; ASD, atrial septal defect; ASA, atrial septal aneurysm; RA, right atrium; COPD, chronic obstructive pulmonary disease; V/Q ratio, ventilation/perfusion ratio. ^1^ Postpneumectomy shunt can be present with or without elevated right atrial pressure.

**Table 2:** Possible criteria for platypnea–orthodeoxia syndrome.

Dyspnea elicited by upright position that disappears with lying position
Orthodeoxia (sPO_2_ < 90% or pO_2_ < 60 mmHg in upright position, normalization in lying position)
Ascertained interatrial communication
Right-to-left shunt

sPO_2_ = oxygen saturation; pO_2_ = partial pressure of oxygen.
